The article "Suppression of long intergenic non-protein coding RNA 1123 constrains lower extremity deep vein thrombosis via microRNA-125a-3p to target interleukin 1 receptor type 1" was retracted in 2026. Reason: concerns about the peer review.

# Suppression of long intergenic non-protein coding RNA 1123 constrains lower extremity deep vein thrombosis via microRNA-125a-3p to target interleukin 1 receptor type 1

**DOI:** 10.1080/21655979.2022.2076496

**Published:** 2022-06-05

**Authors:** Baocai Yang, ZiXiang Zhang

**Affiliations:** a Department of General surgery, The First Affiliated Hospital of Soochow University, Suzhou City, Jiangsu Province, China; b Department of Vascular Surgery, Yancheng First People’s Hospital of Jiangsu Province, Yancheng, Jiangsu Province, China

**Keywords:** Lower extremity deep vein thrombosis, long intergenic non-protein coding RNA 1123 (LINC01123), MicroRNA-125a-3p, interleukin 1 receptor type 1

## Abstract

Lower extremity deep vein thrombosis (LEDVT) is a disorder of venous return caused by abnormal blood clotting. LEDVT can obstruct the lumen and is the third most common vascular disease after cerebrovascular disease and coronary artery disease. LncRNAs are associated with thrombosis and potentially affect the pathogenesis of DVT. However, no studies have reported the effect of LINC01123 on LEDVT. The aim of this study was to investigate the effect of LINC01123 on LEDVT in rats via the miR-125a-3p/interleukin 1 receptor type 1 (IL1R1) axis. Lentiviral vectors that altering LINC01123, miR-125a-3p and IL1R1 expression were pre-injected into the tail vein of rats, and an LEDVT model was established 1 day later. Detection of LINC01123, miR-125a-3p and IL1R1 expression was performed. Inflammatory factors in femoral venous blood, the length and weight of the thrombus, the histomorphological changes were determined in the rat model. The targeting relation of miR-125a-3p with LINC01123 or IL1R1 was verified. The results presented that LEDVT rats expressed high LINC01123 and IL1R1 and low miR-125a-3p expression levels. After silencing LINC01123 or elevating miR-125a-3p, the rate of thrombosis, length and weight of thrombus, and levels of inflammatory factors were reduced. The targeting relation was presented between miR-125a-3p with LINC01123 or IL1R1. Elevating IL1R1 was available to turn around the action of silence of LINC01123 on LEDVT rats. All in all, suppression of LINC01123 restrains LEDVT via miR-125a-3p to target IL1R1.

## Highlights

- LEDVT rats show higher expression of LINC01123 and IL1R1 and lower expression of miR-125a-3p;
- Downregulating LINC01123 or upregulating miR-125a-3p reduced thrombus and inflammation in LEDVT rats;
- There is a targeting relationship between miR-125a-3p and LINC01123 or IL1R1;
- Up-regulation of IL1R1 can reverse the effect of down-regulation of LINC01123 on LEDVT rats;
- Inhibition of LINC01123 inhibits LEDVT by targeting IL1R1 with miR-125a-3p.

## 1. Introduction

Deep venous thrombosis (DVT) is one of the common venous thromboembolic diseases with low cure rate and high postoperative recurrence rate [1]. DVT covers upper extremity deep vein thrombosis and lower extremity deep vein thrombosis (LEDVT), where LEDVT frequently leads to limb loss, abnormal embolism, pulmonary embolism or post-thrombotic syndrome [2]. In China, about 10 million cases are diagnosed with LEDVT annually. LEDVT patients are manifested with local pain, tenderness, edema and swelling of lower limbs, severely impacting the normal life of patients and causing economic burden to the society [3]. The therapy of LEDVT has been advanced greatly, but the molecular mechanism of LEDVT is still uncertain, which extremely limits the screening of diagnostic markers for LEDVT.

Long non-coding RNAs (LncRNAs), a class of endogenous RNAs with over 200 nucleotides in length, basically have no potential to encode proteins and are implicated in almost all biological processes [4]. Numerous studies have illuminated that LncRNA exerts in the occurrence and development of DVT. For instance, LncRNASirt1-AS alleviates DVT via upregulating Sirt1 to stimulate the degradation of Foxo3a [5]. LncRNA GUSBP5-AS accelerates DVT via microRNA (miR)-223-3p/forkhead box O1/Akt pathway to mediate Fibroblast growth factor 2 and matrix metalloproteinase-2/9 [6]. LINC01123, a newly discovered LncRNA, has been testified to perform as an oncogene in multiple human cancers, including endometrial cancer [7], colon cancer [8] and hepatocellular carcinoma [9]. Recently, a study has clarified that LINC01123 expression is elevated in carotid atherosclerosis and it can boost vascular smooth muscle cell proliferation and migration via modulating miR-1277-5p/Krüppel‑like factor 5 axis [10]. Nevertheless, its expression and role in LEDVT remain unknown.

MicroRNA (miRNA), a kind of non-coding single-stranded RNAs, is available to modulate gene at the post-transcriptional level [11]. Numerous researches have elucidated that aberrant miRNA accelerates the occurrence of diseases, covering LEDVT [12]. For instance, elevated miR-103a-3p constrains the development of acute LEDVT [13] and miR-21 boosts thrombosis regression in LEDVT rat models and performs as a latent prognostic marker of LEDVT [14]. A foregoing study has elucidated that miR-125a-3p expression is reduced in patients with atherosclerosis and is available to modulate proliferation and migration of human aortic smooth muscle cells [15]. Nevertheless, its expression and action in LEDVT have not been clarified.

The study was to explore the role and action mechanism of LINC01123 in LEDVT. We hypothesized that LINC01123 affects rat LEDVT via the miR-125a-3p/IL1R1 axis. By establishing an LEDVT rat model, we found for the first time that LINC01123 was up-regulated in LEDVT, and found that down-regulation of LINC01123 inhibited LEDVT by regulating the miR-125a-3p/IL1R1 axis. Our findings may provide a new therapeutic strategy for patients with LEDVT.

## 2. Materials and methods

### 2.1. Construction of LEDVT rat model

Sprague-Dawley (SD) rats (300 ± 20 g) were purchased from Experimental Animal Center of Kunming Medical University (Kunming, Yunnan, China) and fed under specific pathogen free conditions. After adaptation of 2 weeks, an LEDVT rat model was established by blocking femoral veins on both sides under sterile conditions [16]. Rats were anesthesized by intraperitoneal injection of 3% pentobarbital sodium (1 mL/kg, Shanghai Xingzhi Chemical Plant, Shanghai, China) and fixed in a supine position. The skin of the inner thigh was cut lengthwise, the femoral vein was exposed at a depth of 2 cm, and three different sites of the vein were clamped with a mosquito forceps. After establishing the rat model, the incision was sutured. The rats resumed normal eating after regaining consciousness. After 1 day of modeling, the swelling degree of lower limbs and skin color of extremities were observed. The subjects were rats with swollen legs and signs of bruising. Rats in the Sham group were not treated [17].

### 2.2. Rat grouping and lentivirus vector injection

The groups of rats and corresponding treatments are shown (supplementary table S1). One day before modeling, the lentivirus (1 × 10^10^ TU/mL) including sh-negative control (NC), sh-LINC01123, agomir NC, miR-125a-3p agomir, sh-LINC01123 + oe-NC, sh-LINC01123 + oe-interleukin 1 receptor type 1 (IL1R1) was injected into rats through the tail vein. Lentiviral vectors are provided by Thermo Scientific (Open Biosystems, Huntsville, AL) with plasmid and lentiviral packaging systems, high titer lentiviral particles were constructed, packaged and concentrated in the laboratory.

### 2.3. Enzyme-linked immunosorbent assay (ELISA)

The tests were performed in the light of the instructions of the ELISA Kit (eBioscience, San Diego, CA, USA). In short, after 14 d of modeling, femoral vein blood (100 μL) of rats in each group was taken and incubated for 90 min. After that, the sample was incubated with 100 μL fresh biotinylated antibody for 60 min, and added with 100 μL enzyme binding reaction (dark) working solution. After 30 min, the sample was reacted with the substrate (100 μL) for 15 min, and the optical density (OD) was measured at the wavelength of 450 nm on a multifunctional microplate reader (Bio-rad, Hercules, California, USA). Interleukin (IL)-6 and IL-8 were analyzed.

### 2.4. Measurement of thrombus length and weight

After 14 d of modeling, an intraperitoneal injection with 3% pentobarbital sodium was performed on rats for anesthesia. After that, rats were fixed in a supine position on the operating table. The inner thigh skin was then cut longitudinally, the femoral vein was exposed to a depth of 2 cm of the incision, and the femoral vein and thrombus were cut. The weight and length of the thrombus were recorded.

### 2.5. Hematoxylin-eosin (HE) staining

After 14 d of modeling, rats were euthanized by cervical dislocation and the femoral veins were taken, cut, and fixed with 10% neutral formaldehyde solution. After dehydration with 70%, 80%, 90% and 100% ethanol, the samples were treated with xylene, embedded in paraffin, and cut into 4-μm sections. Then, the sections were dewaxed with xylene, hydrated with gradient ethanol (100%, 90%, 80%, 70%), and subjected to HE staining. Next, the sections were dehydrated with ethanol, cleared with xylene, and fixed with neutral balm. The histomorphological changes were observed by optical microscopy (LX51, OLYMPUS, Tokyo, Japan).

### 2.6. Masson staining

Paraffin-embedded tissue sections were dewaxed, stained with Weiger iron-hematoxylin and differentiated with hydrochloric acid ethanol. Next, the sections were stained with ponceau-acidic magenta solution and treated with 1% phosphoric acid aqueous solution for 5 min until the collagen fibers or background became colorless and the myelin sheath was red. Then, the sections were re-stained with aniline blue solution, treated with 1% glacial acetic acid, dehydrated with 95% ethanol and anhydrous ethanol, cleared with xylene and blocked with neutral resin. Finally, sections were observed under an inverted microscope (XSP-8CA, Shanghai Optical Instrument Factory, Shanghai, China) [13].

### 2.7. Reverse transcription quantitative polymerase chain reaction (RT-qPCR)

Extraction of total RNA was implemented using the miRNeasy Mini Kit (Qiagen, Hilden, Germany) in the light of the manufacturer’s instructions. Quantitation of RT-PCR was performed with SYBR Premix Ex Taq (Takara, Japan). PCR was performed in ABI Prism 7900HT rapid real-time PCR system (Applied Biosystems, Life Technologies, USA). U6 or glyceraldehyde-3-phosphate dehydrogenase (GAPDH) was loading control, and the relative quantitative expression was calculated by 2^−ΔΔCt^ method. Primer sequences (GenePharma, Shanghai, China) were presented in Table 1.

**Table 1.** Primer sequences

Genes	Sequences
LINC01123	F: 5’-TTTTGGTTTGAGGGCATAGGG-3’
	R: 5’-CAACAGCATTGACGAGACACATTT-3’
MiR-125a-3p	F: 5’-TGACACAGGTGAGGTTCTTG-3’
	R: 5’-TATGGTTTTGACGACTGTGTGAT-3’
IL1R1	F: 5’-GTGCTACTGGGGCTCATTTGT-3’
	R: 5’-GGAGTAAGAGGACACTTGCGAAT-3’
U6	F: 5’-CGCTTCGGCAGCACATATAC-3’
	R: 5’- AAATATGGAACGCT-TCACGA-3’
GAPDH	F: 5’- ACCCAGAAGACTGTGGATGG-3’
	R: 5’- GGAGACAACCTGGTCCTCAG-3’

### 2.8. Western Blot

Total protein was extracted using Radio-Immunoprecipitation assay lysis buffer containing protease inhibitor (Beyotime Biotechnology, Shanghai, China) and quantified by bicinchoninic acid method. Total protein was separated by 10% sodium dodecyl sulfate-polyacrylamide gel electrophoresis (50 μg/lane) and electroblotted onto a nitrocellulose membrane, and blocked with 5% skim milk. The membrane was incubated with primary antibodies IL1R1 (AB106278) and GAPDH (AB8245) (both 1: 1000, Abcam), and horseradish peroxidase-conjugated secondary antibody. Visualization of protein bands was performed using enhanced chemiluminescence (Pierce; Thermo Fisher Scientific, Inc.). OD was analyzed using Gel Pro analyzer software 4.5 (Beijing Zhongsheng Tiancheng Technology Co., Ltd.).

### 2.9. The luciferase activity assay

The 3ʹuntranslated region fragment of IL1R1 was predicted, and amplified by PCR. Co-transfection of firefly luciferase reporters (LINC01123-wide-type [WT], LINC01123-mutant-type [MUT], IL1R1-WT, IL1R1-MUT), renilla luciferase vector (pMIR-Report Luciferase, Promega) and mimic NC or miR-125a-3p mimic was performed in HEK293T cells according to the instruction of Lipofectamine 2000 (Invitrogen, USA). firefly and renilla luciferase activities were analyzed on a Spectra ™ single tube multimode reader (Sunnyvale, CA, USA).

### 2.10. Statistical analysis

Statistical analysis was implemented using SPSS 21.0 software (IBM, Armonk, NY, USA). Measurement data were expressed as mean ± standard deviation (SD). The two-group comparison was conducted by independent sample *t* test. *P* < 0.05 was accepted with statistical differences.

## 3. Results

### 3.1. LINC01123 and IL1R1 are elevated, while miR-125a-3p is silenced in LEDVT rats

Detection of the histomorphological changes of femoral vein in LEDVT rats and measurement of the length and weight of thrombus were implemented. It was shown that in LEDVT rats, vascular endothelial cells (VECs) were discontinuous, inflammatory cell infiltration around the blood vessels increased, thrombosis in the lumen, and further collagen fibrosis and hyperplasia appeared, some of which entered the thrombus (Figure 1(a-d)). These findings manifested the rat model was successfully established. Inflammatory cytokines IL-6 and IL-8 in the serum of LEDVT rats were elevated (Figure 1(e,f)). Notably, LINC01123 and IL1R1 levels were augmented, while miR-125a-3p level was silenced in LEDVT rats (Figure 1(g,h)). To sum up, LINC01123 and IL1R1 levels were elevated, while miR-125a-3p level was silenced in LEDVT rats.

**Figure 1.** LINC01123 and IL1R1 are elevated while miR-125a-3p is silenced in LEDVT rats. (a): HE staining assessment of pathological conditions; (b): Masson staining evaluation of pathological conditions; (c-d): Length and weight of thrombus; (e-f): Inflammatory cytokines IL-6 and IL-8 in the serum; (g-h): RT-qPCR or Western Blot examination of LINC01123, miR-125a-3p and IL1R1. Values are expressed as mean ± standard deviation (n = 6). * Vs. the Sham, *P* < 0.05.

### 3.2. Repression of LINC01123 constrains inflammation and thrombosis in LEDVT rats

To illuminate the action of LINC01123 in LEDVT, lentivirus sh-NC or sh-LINC01123 was injected into rats. The results clarified that LINC01123 expression declined after injection with sh-LINC01123 (Figure 2(a)). It was observed that thrombus length and weight were reduced after silencing LINC01123 (Figure 2(b,c)) and IL-6 and IL-8 levels in the serum were suppressed (Figure 2(d,e)). After injection with sh-LINC01123, vascular endothelial cells continued to increase, inflammatory cell infiltration, intraluminal thrombosis, and collagen fiber proliferation decreased in LEDVT rats (figure 2(f,g))). In brief, silence of LINC01123 restrained inflammation and thrombosis in LEDVT rats.

**Figure 2.** Silence of LINC01123 represses inflammation and thrombosis in LEDVT rats. (a): RT-qPCR test of LINC01123; (b-c): Length and weight of thrombus; (d-e): Inflammatory cytokines IL-6 and IL-8 in the serum; (f): HE staining assessment of pathological conditions; (g): Masson staining evaluation of pathological conditions; Values are expressed as mean ± standard deviation (n = 6). * Vs. the sh-NC, *P* < 0.05.

### 3.3. LINC01123 modulates IL1R1 via miR-125a-3p

It was testified that LINC01123 and IL1R1 levels were augmented, while miR-125a-3p level was silenced in LEDVT rats, so the targeting relation was predicted between miR-125a-3p with LINC01123 or IL1R1. It was discovered that targeted binding sites were presented between miR-125a-3p with LINC01123 or IL1R1 (Figure 3(a,b)). Luciferase activity was impaired after co-transfection with LINC01123-WT or IL1R1-WT and miR-125a-3p mimic (Figure 3(c,d)). Additionally, after silencing LINC01123, miR-125a-3p level was augmented, while IL1R1 level was decreased (Figure 3(e,f)). In general, LINC01123 modulated IL1R1 via miR-125a-3p.

**Figure 3.** LINC01123 modulates IL1R1 via miR-125a-3p. (a-b): Bioinformation website prediction of the targeted binding site of miR-125a-3p with LINC01123 or IL1R1; (c-d): The luciferase activity assay verification of the targeting of miR-125a-3p with LINC01123 or IL1R1; E-F: RT-qPCR or Western Blot detection of miR-125a-3p with IL1R1. Values are expressed as mean ± standard deviation (n = 6), cell experiments were repeated three times. * Vs. the sh-NC, P < 0.05.

### 3.4. miR-125a-3p represses inflammation and thrombosis in LEDVT rats

To explore the action of miR-125a-3p in LEDVT, lentivirus agomir NC or miR-125a-3p agomir was injected into rats. miR-125a-3p agomir resulted in the upregulation of miR-125a-3p in rats (Figure 4(a)), which beneficially decreased the length and weight of thrombus (Figure 4(b,c)), levels of IL-6 and IL-8 in the serum (Figure 4(d,e)), and alleviated the histopathology of femoral vein in LEDVT rats (figure 4(f,g)). In brief, miR-125a-3p restrained inflammation and thrombosis in LEDVT rats.

**Figure 4.** Elevated miR-125a-3p represses inflammation and thrombosis in LEDVT rats. (a): RT-PCR test of miR-125A-3p; (b-c): Length and weight of thrombus; (d-e): Inflammatory cytokines IL-6 and IL-8 in the serum; (f): HE staining assessment of pathological conditions; (g): Masson staining evaluation of pathological conditions; Values are expressed as mean ± standard deviation (n = 6). * Vs. the agomir NC group, *P* < 0.05.

### 3.5. Elevated IL1R1 turns around the action of silenced LINC01123 on LEDVT rats

To further verify the role of LINC01123 in LEDVT via modulating miR-125a-3p/IL1R1 axis, rats were injected with lentivirus sh-LINC01123 + oe-NC or sh-LINC01123 + oe-IL1R1. oe-IL1R1 reversed sh-LINC01123-mediated downregulation of IL1R1 (Figure 5(a)), resulting in increased thrombus length and weight (Figure 5(b,c)), elevated IL-6 and IL-8 levels in the serum (Figure 5(d,e)), and aggravated histopathology of femoral vein (figure 5(f,g)). All in all, elevated IL1R1 turned around the action of suppression of LINC01123 on LEDVT rats.

**Figure 5.** Elevated IL1R1 turns around the action of repressive LINC01123 on LEDVT rats. (a): RT-qPCR and Western Blot verification of successful injection; (b-c): Length and weight of thrombus; (d-e): Inflammatory cytokines IL-6 and IL-8 in the serum; F: HE staining assessment of pathological conditions; (g): Masson staining evaluation of pathological conditions; Values are expressed as mean ± standard deviation (n = 6). * Vs. the sh-LINC01123 + oe-NC, *P* < 0.05.

## 4. Discussion

LEDVT is the third critical cardiovascular disease after cerebrovascular disease and coronary artery disease [18]. As reported, injury and dysfunction of VECs are crucial factors in the occurrence of LEDVT [19]. LncRNAs are implicated in multiple cardiovascular diseases covering LEDVT via mediating the cellular process of VECs [20]. In this research, it was testified that LINC01123 expression was elevated in LEDVT rats, and silenced LINC01123 distinctly reduced the length and weight of thrombus, levels of IL-6 and IL-8 in the serum, constrained inflammatory cell infiltration, thrombosis in the lumen and collagen fiber hyperplasia. These results suggested that LINC01123 was as a novel pathogenic factor of LEDVT and offered a brand-new latent target for the treatment of LEDVT.

Antecedent studies have elaborated that LINC01123 is elevated in multiple types of cancer and performs as an oncogene. For instance, LINC01123 accelerates proliferation and aerobic glycolysis of non-small cell lung carcinoma via miR-199a-5p/c-Myc axis [21]. Elevated LINC01123 forebodes the poor prognosis of oral squamous cell carcinoma (OSCC) and modulates OSCC cell growth via absorbing miR-34a-5p [22]. The action of LINC01123 in cancer has been explicit, but its role in LEDVT is uncertain. Numerous studies have illuminated that the interaction is presented between thrombosis and inflammation, and DVT is linked with the aggravation of inflammation at diagnosis [23]. Consequently, inflammation might be either a cause or a result of DVT. In this study, a rat model of LEDVT was established in rats, and it was discovered that were discontinuous, inflammatory cell infiltration around the blood vessels increased, thrombosis in the lumen, and further collagen fibrosis and hyperplasia appeared, some of which entered the thrombus, and inflammatory cytokines IL-6 and IL-8 in the serum were elevated in rats after surgery. These results elaborated that the LEDVT rat model was successfully constructed and confirmed that LEDVT was associated with inflammation. Additionally, LINC01123 expression was elevated in LEDVT rats, while silence of LINC01123 restrained inflammation and thrombosis in LEDVT rats. LncRNAs perform as a competitive endogenous RNAs (ceRNA) of miRNAs, thus mediating downstream target genes of miRNA [24]. LINC01123 is available to act as a sponge for multiple miRNAs, like miR-625-5p [25] and miR-151a, etc [26]. In this study, the downstream targets of LINC01123 were further explored. It was testified that LINC01123 modulated miR-125a-3p.

miRNAs are dysregulated in diversified human illnesses and perform as circulating biomarkers for certain cardiovascular diseases, covering LEDVT [13], atherosclerosis [27] and abdominal aortic aneurysm [28]. Foregoing researches have clarified that miR-125a-3p is silenced in hemangioma (HA), while elevated miR-125a-3p constrains the proliferation, migration and invasion of HA-derived endothelial cells [29]. MiR-125a-3p is silenced in restenosis arteries after vascular interventional therapy of lower extremity, and effectively represses vascular smooth muscle cell (VSMCs) function and the occurrence of vascular stenosis via targeting mitogen-activated protein kinase 1 [30]. Recently, a study has manifested that miR-125a-3p is silenced in patients with carotid atherosclerosis, while elevated miR-125a-3p represses cell viability, cell cycle progression and migration of human aortic VSMCs [15]. In this research, it was discovered that miR-125a-3p was silenced in LEDVT rats, while elevated miR-125a-3p reduced the length and weight of thrombus as well as IL-6 and IL-8 in the serum and ameliorated the histopathology of femoral vein in LEDVT rats. As known, this was the first report to explicitly indicate the action of miR-125a-3p in LEDVT.

IL1R1 is a cytokine receptor that belongs to the IL-1 receptor family, and is available to modulate cell metabolism and multiple cytokine-induced immune inflammatory responses [31]. IL1R1 exerts a critical role in LEDVT and its expression could be modulated by miRNA [32]. In this research, IL1R1 is elevated in LEDVT rats and its expression was mediated by miR-125a-3p. Additionally, augmented IL1R1 was available to turn around the action of repression of LINC01123 or elevation of miR-125a-3p. These results manifested that LINC01123/miR-125a-3p/IL1R1 axis exerted a critical role in LEDVT.

## 5. Conclusion

In brief, the study has testified that LINC01123 is upregulated in LEDVT and is a novel biomarker of LEDVT. LINC01123 increases thrombus length and weight in LEDVT rats by regulating the miR-125a-3p/IL1R1 axis, increases serum IL-6 and IL-8 levels, inhibits VEC proliferation, and increases inflammatory cell infiltration, intraluminal thrombosis, collagen fibers and hyperplasia, which in turn promote inflammation and thrombosis in LEDVT rats. The research results might offer novel treatments for LEDVT patients.

## Supplementary Material

Supplemental Material
